# Efficacy of Dapagliflozin in Patients with Diabetes Mellitus Complicated with Coronary Artery Disease and Its Impact on the Vascular Endothelial Function

This article has been retracted.

**DOI:** 10.1155/2022/4829750

**Published:** 2022-09-09

**Authors:** Fei Ma, Jun Zhang, Huan Wang, Yan Wu, Yuliang Wu

**Affiliations:** ^1^Cardiovascular Department, The Central Hospital of Tongchuan Mining Bureau, Tongchuan, China; ^2^Cardiovascular Department, The First Affiliated Hospital of Xi'an Jiaotong University, Xi'an, China

## Abstract

**Objective:**

To investigate the efficacy of dapagliflozin for diabetes mellitus complicated by coronary artery diseases and its impact on vascular endothelial function.

**Methods:**

Between August 2020 and August 2021, 80 patients with coronary heart disease complicated by type 2 diabetes mellitus were recruited and randomly assigned to receive either dapagliflozin (5 mg daily) plus original oral hypoglycemic agents (dapagliflozin group) or original oral hypoglycemic agents alone (control group). Outcome measures included blood pressure, blood glucose, cholesterol levels, vascular endothelial function, cardiovascular events, and drug-related adverse events.

**Results:**

The two groups had similar outcome indices upon admission (*P* > 0.05). After 20 weeks of medication, the two groups of patients showed similar blood pressure, hemoglobin A1c (HbA1c), and low-density lipoprotein (LDL-C) levels versus those before treatment (*P* > 0.05), and no significant differences were found in intergroup comparison neither (*P* > 0.05). Dapagliflozin plus conventional hypoglycemic agents resulted in a significantly higher reactive hyperemia index (RHI) value, fewer cases with abnormal vascular endothelial function, and fewer major cardiovascular events during treatment versus the sole use of conventional hypoglycemic agents (*P* < 0.05). There was no significant difference in drug-related adverse events between the two groups (*P* > 0.05).

**Conclusion:**

Dapagliflozin improves the vascular endothelial functions of patients with diabetes mellitus complicated by coronary artery disease with a high safety profile and favorable efficacy.

## 1. Introduction

Type 2 diabetes mellitus is a major risk factor for cardiovascular disease. Several new antidiabetic drugs have been developed clinically, which have also shown good cardiovascular protection. The DAPA-HF study showed that dapagliflozin reduced cardiovascular and all-cause mortality in patients with heart failure with reduced ejection fraction, regardless of the comorbidity of type 2 diabetes mellitus. Concurrently, the hypertensive disease is a common comorbidity of type 2 diabetes mellitus. Numerous studies have shown that diabetic patients with comorbid hypertension are at higher cardiovascular risk compared to diabetic patients without comorbid hypertension. Coronary heart disease is a common complication in diabetic patients, and disease progression may result in more clinical adverse events. And glycemic management is crucial for the prevention and treatment of vascular disease progression in these patients [1, 2].

Recent studies have revealed a significant role of abnormal endothelial function in the development of vascular diseases such as coronary artery disease. Recent studies suggest that abnormal endothelial function may be one of the nontraditional risk factors for coronary heart disease and independent of traditional risk factors such as age, blood pressure, and lipids and may predict adverse cardiovascular events and myocardial infarction size. Type 2 diabetes is characterized by inadequate or resistant insulin production, whereas coronary heart disease is caused by coronary artery sclerosis, with symptoms such as angina pectoris. The increased incidence of type 2 diabetes mellitus caused by coronary artery disease severely compromises the quality of life of patients.

Dapagliflozin is a class of hypoglycemic agents that has received considerable attention in recent years [3, 4]. It lowers blood glucose and blood pressure, ameliorates blood lipids, and provides cardioprotective effects [5]. It effectively reduces the reabsorption of glucose by the kidneys, thereby lowering the patient's blood glucose concentration. In addition, there is an additional benefit of reduced blood pressure levels, which may be attributable to its natriuretic and diuretic effects. However, it is not clear whether these benefits can also be observed in the Chinese population. The present study was conducted to investigate the efficacy of dapagliflozin in patients with diabetes mellitus complicated with coronary artery disease and its impact on the vascular endothelial function, to provide more basis for the clinical application of dapagliflozin.

## 2. Materials and Methods

### 2.1. Participants and Grouping

Between August 2020 and August 2021, 80 patients with coronary heart disease complicated by type 2 diabetes mellitus were recruited and randomly assigned to receive either dapagliflozin (5 mg daily) plus original oral hypoglycemic agents (dapagliflozin group) or original oral hypoglycemic agents alone (control group). The diagnosis criteria followed the Chinese Medical Association's norms. The baseline statistics for the two groups were comparable (*P* > 0.05) (Table 1).

The randomization was carried out using an online web-based randomization tool (freely available at http://www.randomizer.org/). For concealment of allocation, the randomization procedure and assignment were managed by an independent research assistant who was not involved in the screening or evaluation of the participants.

For sample size calculation, the sample size was determined according to the hospital sampling survey case-control study method, the estimated prevalence was 5%, the relative error of the sampling survey was 20% and set at 1.5, with a 95% confidence interval, *Za* = 1.96 and a 10% data incompleteness rate, and the final calculated sample size was in the range of 35 to 50.

The trial was done in accordance with the standards of Good Clinical Practice and the Declaration of Helsinki. The trial protocol and all amendments were approved by the appropriate ethics body at each participating institution. All patients provided written informed consent before enrolment. The trial protocol has been published online and is available with the full text of this article. Ethics number is as follows: HU-TY20200708.

Inclusion criteria are as follows: (1) aged ≥60 years; (2) with the current use of dapagliflozin tablets (concomitant use of insulin is available), with a treatment duration of ≥5 months; (3) with current oral administration of non-SGLT2 inhibitor hypoglycemic drugs (can use insulin at the same time); (4) age ≥ 18 years; and (5) with fasting blood glucose (FBG) ≤ 10 mmol/L and glycosylated hemoglobin (HbAlc) ≤ 8.5%.

Exclusion criteria are as follows: (1) patients with severe heart failure (cardiac insufficiency grades III-IV); (2) with acute myocardial infarction; (3) with liver and kidney insufficiency; (4) with acute and chronic infections, hematological diseases, malignant tumors, rheumatic connective tissue, and other immune system diseases; (5) with recent surgery or trauma; and (6) with a bodyweight of <50 kg.

### 2.2. Treatment Methods

#### 2.2.1. Dapagliflozin Group

Oral dapagliflozin (5 mg daily) was added on top of the original oral hypoglycemic drugs, and the original oral hypoglycemic drugs could be reduced or discontinued depending on the blood glucose level of the patients.

#### 2.2.2. Control Group

The initial oral hypoglycemic medicines were continued, and the dose could be modified based on the patients' blood glucose levels. Except for extreme adverse responses, all patients were treated for 20 weeks until the completion of the study. In both groups, the secondary preventive medicine for coronary heart disease remained unchanged.

### 2.3. Outcome Measures

#### 2.3.1. Blood Pressure, Blood Glucose, and Blood Lipid Levels

Blood pressure, glycosylated hemoglobin (HbA1c), and low-density lipoprotein (LDL-C) levels were compared between the two groups upon admission and after 20 weeks of treatment.

The blood pressure was measured, and morning fasting venous blood was obtained from the patient at 7 : 00 on the day before and the day after the treatment in both groups: (1) HbAlc: high-performance liquid chromatography (HPLC) was performed using an HA-8180 HbAlc analyzer and original reagents. (2) LDL-C: the Japanese Sekisui Surfactant Removal (SUR) method was used to determine the LDL-C using the SP-4430 biochemistry analyzer and original reagents.

#### 2.3.2. Vascular Endothelial Function

The values of the vascular endothelial function at admission and after 20 weeks of treatment and the cases of abnormalities in vascular endothelial function were compared between the two groups. Reactive hyperemia index (RHI), which reflects nitric oxide-dependent changes in endothelial function, was obtained using the EndoPAT-2000 Itamar assay, and abnormal vascular endothelial function was determined by an RHI < 1.67. The patient fasted for 4 hours prior to the test, which was conducted in a calm, temperature-controlled environment with consistent illumination. The EndoPAT-2000 finger cuffs were put on the subject's two middle fingers, and pressure changes in the cuffs caused by pulsatile volume changes in the distal fingers were detected by a pressure sensor and communicated to the Endo-PAT device for recording. RHI testing: The baseline measurement was performed for 5 min, after which the blood pressure cuff on the test arm was inflated to 60 mmHg above the baseline systolic pressure, and blood flow was blocked for 5 min, followed by deflation of the cuff and recording for another 6 min after deflation.

#### 2.3.3. Cardiovascular Events

The incidence of major cardiovascular events (angina pectoris, myocardial infarction, heart failure, and cardiac death) within 20 weeks was recorded and compared between the two groups.

#### 2.3.4. Adverse Drug Events

The incidence of drug-related adverse events such as hypoglycemia, severe hypoglycemia, hypotension (blood pressure < 90/60 mmHg), and wasting (weight loss with a weight of less than 10% of standard body weight) were recorded and compared between the two groups within 20 weeks.

### 2.4. Statistical Analysis

The mean difference between the two groups was tested using the Student *t*-test for normally distributed variables and the Mann-Whitney *U* test for nonnormal variables. SPSS 18.0 was used for data analyses. The measurement data were expressed as *x̅*±*s* and processed using the *t*-test. The count data were expressed as the number of cases (rate) and analyzed using the chi-square test. Differences were considered statistically significant at *P* < 0.05.

## 3. Results

### 3.1. Blood Pressure, HbA1c, and LDL-C Levels

The two groups had similar outcome indices upon admission (*P* > 0.05). After 20 weeks of medication, the two groups of patients showed similar blood pressure, HbA1c, and LDL-C levels versus those before treatment (*P* > 0.05) (Table 2).

### 3.2. Vascular Endothelial Function

Before treatment, the difference in the RHI values and cases with abnormal vascular endothelial function did not come up to the statistical standard (*P* > 0.05). Dapagliflozin plus standard hypoglycemic medications resulted in considerably higher RHI values and fewer instances with impaired vascular endothelial function (RHI < 1.67) (*P* < 0.05) (Table 3).

### 3.3. Cardiovascular Events

Dapagliflozin plus conventional hypoglycemic agents was associated with fewer major cardiovascular events during treatment versus the sole use of conventional hypoglycemic agents (*χ*^2^ = 4.39; *P* < 0.05) (Table 4).

### 3.4. Drug-Related Adverse Events

Each group experienced two hypoglycemic responses, but no severe hypoglycemia, hypotension, or wasting episodes occurred. Three instances in the dapagliflozin group had lower blood pressure than before the treatment, and dapagliflozin was maintained after antihypertensive medicines were reduced appropriately. There was no significant difference between the two groups in terms of drug-related adverse events (*P* > 0.05).

## 4. Discussion

The 7th edition of the International Diabetes Federation (IDF) Diabetes Map shows that 415 million adults worldwide had diabetes in 2015, and by 2040, more than 640 million adults are diagnosed with diabetes. Data show that 75% of type 2 diabetic patients die from cardiovascular disease. Coronary artery lesions in type 2 diabetic patients are prevalent as subtle, diffuse, calcified, and multivessel lesions, and there is a high incidence of stent restenosis and hemodynamic reconstitution in type 2 diabetic patients after PCI. Glycemic management is a therapeutic priority for patients with coronary artery disease with underlying diabetes mellitus [6, 7]. Traditional oral hypoglycemic agents are mainly used to reduce cardiovascular risk by blood glucose control, and only metformin may provide additional cardiovascular benefits. The novel hypoglycemic agent sodium-glucose cotransport protein 2 (SGLT-2) inhibitor inhibits glucose reabsorption by the proximal tubular SGLT family, thereby reducing blood glucose levels. In addition to hypoglycemia, dapagliflozin is a new type of glucose-lowering medicine that has been developed in recent years, with the benefits of reducing blood pressure, improving blood lipids, and decreasing uric acid. International multicenter clinical trials, such as EMPA-REG and DECLARE, have recently demonstrated that dapagliflozin could lower the risk of cardiovascular events in individuals with diabetes and coronary heart disease and provide cardioprotective benefits [8].

The results of the present study showed that the combined use with dapagliflozin resulted in a lower incidence of angina and heart failure events versus conventional hypoglycemic agents after 20 weeks of treatment, suggesting the priority of dapagliflozin for glucose-lowering therapy in patients with diabetes mellitus combined with coronary artery disease. Abnormalities in vascular endothelial function appear early in the course of the vascular-related disease and persist throughout. SGLT2i increases urinary glucose excretion, and the osmotic diuretic and natriuretic effects due to increased urinary glucose contribute to a reduction in blood volume, with patients experiencing a reduction in systolic and diastolic blood pressure of 4-6 mmHg and 1-2 mmHg, respectively, which underlies potential cardiovascular benefits.

Recent studies have demonstrated that abnormal vascular endothelial function may be one of the nontraditional risk factors for coronary heart disease and independent of traditional risk factors, such as age, blood pressure, and blood lipids, and may predict adverse cardiovascular events and myocardial infarction size [9–13]. The RHI is an established indicator of vascular endothelial function. The present study found that abnormal endothelial function (RHI < 1.67) was still found in about 40% of the elderly population with diabetes mellitus complicated by coronary artery disease; most of whom were treated with related medications, which indicates the modest effects of conventional drugs on the improvement of vascular endothelial function [14–17]. Moreover, dapagliflozin herein was associated with fewer patients with abnormal RHI after treatment, which is suggestive of the benefits of dapagliflozin in vascular endothelial function [18–20].

The present study also revealed an overall increase in RHI values in the dapagliflozin group and fewer cardiovascular events versus the patients in the control group, indicating that dapagliflozin is effective in improving vascular endothelial function, and the improvement of vascular endothelial function is speculated to be a contributor to the reduction of cardiovascular events. The absence of significant differences in the adverse events between the two groups indicates a high safety profile of dapagliflozin. Nevertheless, the occurrence of occasional hypoglycemic reactions requires close monitoring of blood glucose for drug changes. It is hypothesized that SGLT2 may inhibit oxidative stress and inflammatory responses in the vascular endothelium, optimize cardiomyocyte energy metabolism, and improve hemodynamics through inhibitors, but the specific mechanisms by which it improves vascular endothelial function remain to be explored [21].

As an SGLT-2 inhibitor, dapagliflozin improves clinical outcomes in coronary artery disease through multiple mechanisms. First, dapagliflozin has good glycemic control. The results of several large multicenter clinical studies showed that dapagliflozin significantly reduced glycated hemoglobin, fasting glucose, and postprandial glucose [22]. Second, dapagliflozin controls blood pressure. One study found that dapagliflozin reduced systolic blood pressure by a mean of 11.9 mmHg (1 mmHg = 0.133 kPa). Third, dapagliflozin controls weight. Dapagliflozin was unexpectedly found to reduce patients' weight during the follow-up of clinical studies, thanks to dapagliflozin's ability to excrete more glucose from the body and reduce body fat (visceral fat, subcutaneous fat, and total fat) [23]. Fourth, dapagliflozin controls inflammation. Through in vitro studies, SGLT-2 inhibitors were found to reduce infarct size and improve cardiac function in reperfused ischemic hearts by inhibiting inflammatory factors and oxidative stress during ischemic episodes [24, 25].

The present experiment has many shortcomings. First, the study sample size was small, the follow-up period was short, and the length of observation was insufficient for such a complex mechanism of change as ventricular remodeling. Ultrasonographic observables were unavailable to observe functional improvement, and therefore, no more structural corroboration was available. In the process of reconstructing the control variables by observation, insufficient monitoring led to certain fluctuations in blood glucose and blood pressure of individual patients during the treatment process, which had an impact on the final results as an influencing factor. Subsequent studies will refine and improve the experimental shortcomings, expand the sample size, extend the observation time, increase the observation index, control the influencing factors, and eliminate the drawbacks, so as to produce more accurate research results. In some current basic and clinical studies, a growing number of possible pathways and biomarkers affecting ventricular remodeling are being confirmed, providing more potential targets for drug research and indicating the direction of exploration to improve the prognosis of patients with cardiovascular disease. In the future, more novel drugs against inhibition of ventricular remodeling and improvement of patient's quality of life can be developed based on such studies, providing more possibilities for clinical treatment.

To sum up, dapagliflozin reduces the incidence of all-cause mortality and cardiovascular death in coronary artery disease combined with type 2 diabetes but fails to lower the incidence of nonfatal myocardial infarction, stroke, revascularization, and readmission. Despite its safety in improving vascular endothelial function in patients, the exact mechanism of dapagliflozin remains unclear.

## Figures and Tables

**Table 1:** Comparison of baseline data.

Indices	Control group (*n* = 40)	Dapagliflozin group (*n* = 40)	*t*/*χ*^2^ value	*P* value
Age (years, *x* ± *s*)	68.30 ± 9.60	69.80 ± 8.20	0.85	0.36
Gender (male, *n*, %)	27 (80.00)	26 (85.72)	0.14	0.66
BMI (kg/m^2^, *x* ± *s*)	23.20 ± 2.30	22.50 ± 2.10	0.58	0.43
Duration of diabetes mellitus (years, *x* ± *s*)	6.90 ± 5.70	7.52 ± 4.68	0.42	0.52
Combined insulin (*n*, %)	5 (16.59)	7 (23.40)	0.43	0.51
Oral hypoglycemic drugs (*n*, %)				
Metformin	11 (35.48)	12 (38.50)	0.08	0.76
Sulfonylurea	12 (39.60)	10 (29.20)	0.28	0.58
Alpha-glucosidase inhibitors	7 (22.90)	9 (29.00)	0.34	0.57
DPP4 inhibitors	8 (25.87)	6 (10.50)	0.36	0.55
Coronary heart disease drugs (*n*, %)				
Antiplatelet agents	30 (100.00)	30 (100.00)	0.01	1.05
Statin	29 (68.40)	27 (70.80)	0.23	0.62
Beta-blockers	13 (42.50)	16 (50.40)	0.58	0.42
ACEI/ARB	14 (68.50)	12 (38.66)	0.28	0.62

**Table 2:** Comparison of blood pressure, HbA1c, and LDL-C levels (*x̅*±*s*).

Indices	Control group (*n* = 40)	Dapagliflozin group (*n* = 40)	*t* value	*P* value
Systolic blood pressure (mmHg)				
Upon admission	125.86 ± 12.92	128.8614.24	22.387	0.49
After 20 weeks of treatment	127.68 ± 13.97	126.0813.15	30.301	0.78
Diastolic blood pressure (mmHg)				
Upon admission	68.78 ± 9.58	71.26 ± 10.84	38.021	0.96
After 20 weeks of treatment	68.96 ± 10.08	70.76 ± 11.06	20.896	1.16
HbA1c (%)				
Upon admission	6.86 ± 0.88	7.16 ± 1.14	51.056	0.83
After 20 weeks of treatment	6.80 ± 1.04	6.96 ± 1.24	69.058	0.94
LDL-C (mm01/L)				
Upon admission	2.32 ± 0.84	2.43 ± 0.72	40.340	0.06
After 20 weeks of treatment	2.28 ± 0.68	2.30 ± 0.83	43.321	0.01

**Table 3:** Comparison of vascular endothelial function.

Indices	Control group (*n* = 40)	Dapagliflozin group (*n* = 40)	*t* value	*P* value
RHI value (*x̅*±*s*)				
Upon admission	1.76 ± 0.31	1.81 ± 0.36	7.232	0.475
After 20 weeks of treatment	1.77 ± 0.33	1.88 ± 0.37	9.023	0.023
RHI < 1.67 (*n*,%)				
Upon admission	13 (42.96)	12 (39.98)	11.378	0.798
After 20 weeks of treatment	12 (39.98)	5 (15.88)	11.208	0.044

**Table 4:** Comparison of cardiovascular events (*n*, %).

Cardiovascular events	Control group (*n* = 40)	Dapagliflozin group (*n* = 40)	*χ* ^2^	*P* value
Angina pectoris	8 (22.32)	3 (12.66)		
Myocardial infarction	1 (3.24)	1 (3.24)		
Heart failure	4 (9.98)	1 (2.13)		
Cardiac death	0 (0.00)	0 (0.00)		
Total incidence	13 (35.54)	5 (18.03)	4.39	0.023

## Data Availability

All data generated or analyzed during this study are included in this published article.
